# Improved Machine Learning Method for Intracranial Tumor Detection with Accelerated Particle Swarm Optimization

**DOI:** 10.1155/2022/1128217

**Published:** 2022-03-03

**Authors:** K. R. Pradeep, Syam Machinathu Parambil Gangadharan, Wesam Atef Hatamleh, Hussam Tarazi, Piyush Kumar Shukla, Basant Tiwari

**Affiliations:** ^1^Department of Computer Science & Engineering, B.M.S Institute of Technology and Management, Avalahalli, Bengaluru 560064, India; ^2^General Mills, 220 Carlson Parkway, Apt 208, Minnetonka 55305, Minnesota, USA; ^3^Department of Computer Science, College of Computer and Information Sciences, King Saud University, P.O. Box 51178, Riyadh 11543, Saudi Arabia; ^4^Department of Computer Science and Informatics, School of Engineering and Computer Science, Oakland University, Rochester Hills, 318 Meadow Brook Rd, Rochester 48309, MI, USA; ^5^Department of Computer Science & Engineering, University Institute of Technology, Rajiv Gandhi Proudyogiki Vishwavidyalaya, Bhopal 462033, Madhya Pradesh, India; ^6^Department of Computer Science, Hawassa University, Awasa, Ethiopia

## Abstract

The field of image processing is distinguished by the variety of functions it offers and the wide range of applications it has in biomedical imaging. It becomes a difficult and time-consuming process for radiologists to do the manual identification and categorization of the tumour. It is a complex and time-consuming procedure conducted by radiologists or clinical professionals to remove the contaminated tumour region from magnetic resonance (MR) pictures. It is the goal of this study to improve the performance and reduce the complexity of the image segmentation process by investigating FCM predicted image segmentation procedures in order to reduce the intricacy of the process. Furthermore, relevant characteristics are collected from each segmented tissue and aligned as input to the classifiers for autonomous identification and relegation of encephalon cancers in order to increase the accuracy and quality rate of the neural network classifier. An evaluation, validation, and presentation of the experimental performance of the suggested approach have been completed. A unique APSO (accelerated particle swarm optimization) based artificial neural network model (ANNM) for the relegation of benign and malignant tumours is presented in this study effort, which allows for the automated identification and categorization of brain tumours. Using APSO training to improve the suggested ANNM model parameters would give a unique method to alleviate the stressful work of radiologists performing manual identification of encephalon cancers from MR images. The use of an APSO-based ANNM (artificial neural network model) model for automated brain tumour classification has been presented in order to demonstrate the resilience of the classification model. It has been suggested to utilise the improved enhanced fuzzy *c* means (IEnFCM) method for image segmentation, while the GLCM (gray level co-occurrence matrix) feature extraction approach has been employed for feature extraction from magnetic resonance imaging (MR pictures).

## 1. Introduction

In the current medical sciences and clinical research developments, many models have been developed for earlier tumor detection for saving a patient's life. Perhaps, detecting tumor from MRI scans is a very time-consuming and complicated process. It takes several times for segmenting the tumor cells from brain tissues [1]. Consequently, image processing techniques have been incorporated for the tumor detection process in recent times, which provides the results faster [2]. Moreover, a brain tumor can be categorized into primary and secondary, further denoted as benign and malignant. Malignant tumors are dangerous that can spread to other parts of the body. So, when the cancer is detected at the benign or initial stages, it can be easily treated by clinical practitioners [3].

The supratentorial cortex is a term used to describe the cortex in specific cases. Located in the frontal lobe of the brain, it is responsible for decision-making. Hemispheres are found on each side of the brain, with one on each side of the brain. It is the cerebrum's responsibility to perform the following activities, among others: movement initiation and coordination, temperature, touch, vision, hearing, judgement, thinking, problem solving, emotions, and learning. The cerebrum, also known as the cortex, is the most important region of the human brain. It is responsible for the majority of cognitive functions. It has been shown to be associated with higher order brain activity such as thinking and action, among other things. The cerebral cortex is divided into four areas, known as lobes, which are as follows: the frontal lobe, the parietal lobe, the occipital lobe, and the temporal lobe. The frontal lobe is the largest of the four lobes. In terms of prominence, the frontal lobe is the most prominent of them. The frontal lobe is engaged in problem solving and critical thinking, among its many other activities. It also regulates a variety of aspects of the voice, movement, and emotions. Parietal lobe regulates the functions of movement, direction, recognition, and perception of inputs in addition to other activities. The occipital lobe is a part of the brain that is involved in the processing of visual information. Aspects of the temporal lobe's function include the detection and identification of auditory events, as well as the storage and creation of words.

Tumor is a standout amongst the most well known and deadly of the regular brain disorders, and it is notably harmful in children. Worldwide, according to estimates, more than four lakh individuals suffer from tumours each year, and early identification and treatment are crucial for more than four lakh people who suffer from tumours each year in the United States. Therapies using imaging technologies have progressed to the point that they may be employed in a variety sectors of medicine, including computer-aided pathology diagnosis, surgical planning, and directing, as well as longitudinal investigation, among others. In neuro-science and neurosurgery, magnetic resonance imaging (MRI) and computed tomography (CT) are the two therapeutic imaging modalities that are most often employed, out of all the therapeutic imaging modalities available. The segmentation of objects from magnetic resonance imaging, especially anatomical structures and disorders, is an important endeavour since the results are extensively utilised as the basis for a range of applications. Segmentation techniques differ significantly based on the specific application and image modality that is being utilised in the segmentation procedure. Additionally, medical image segmentation is a difficult procedure since medical pictures often include a large amount of data as well as a few artefacts as a result of the patient's short collecting period and sensitive tissue boundaries that are not always clearly defined. When dealing with brain tumours, a range of complications arise, making it difficult to categorise them into discrete categories. Various tumour types exist, with each having a distinct mix of forms and sizes. Cancer is classified into several categories. Depending on the scenario, it may emerge in any area and with varied image intensities, or it may occur at all. Some of them induce deformation of the surrounding structures, while others may be connected with oedema, which causes the intensities of pictures around the tumour to change. Oedema is a condition in which the intensity of images around the cancer changes. Additional to this, the existence of a few distinct magnetic resonance imaging collecting methodologies gives various information on the brain's structure and function. With each shot, a different aspect of the tumour is brought to light in some manner. Automatic segmentation based on past models and the utilisation of prior knowledge are both difficult tasks to complete. The exact segmentation of the inner architecture of the brain is a source of considerable interest in both cancer research and the treatment of malignancies, and it is becoming more important. The mortality rate for thyroid cancer is being lowered, and the surgical and radiotherapeutic treatment of thyroid tumours is being improved. An evocative human brain model is also desirable because it enables researchers to coordinate tumour information extracted from magnetic resonance imaging (MRI) and computed tomography (CT) images, such as tumour localization and shape, function, and the tumor's impact on surrounding neural tissue and brain structures, with information extracted from other sources. While the medical imaging industry has made multiple efforts and witnessed some hopeful results in recent years, reliable and repeatable segmentation and abnormalities characterisation continue to be very difficult tasks. Automation, applicability, and accuracy are all areas where existing approaches have significant space for improvement. Because it can image at any angle without the use of potentially harmful radiation, magnetic resonance imaging (MRI) is excellent for diagnosing diseases of large vessels as well as structural changes of the heart and heart lining. It also provides more accurate information than conventional echocardiogram regarding the structure and function of the heart, as well as excellent tissue differentiation regardless of whether contrast material is used. The MRI system may cause tissues in the body to appear in a number of different ways depending on the examination settings that are used during the procedure. This is quite beneficial in judging if anything seen is normal or abnormal. The disadvantages of magnetic resonance imaging (MRI) are the lengthy study time necessary, the loud noises generated, and the restricted setting in which it must be performed. Additional limitations include the presence of some metallic biomedical equipment or foreign objects that prevent MRI from being conducted.

There different kinds of brain tumor diagnosis methodologies are developed in the recent decade. In general, the automatic tumor segmentation issues are complicated, and new inventions are still required to solve problems. Moreover, the processing functions include typical operations such as image preprocessing, tissue segmentation, feature extraction, and image classifications.  Figure 1 displays the pictorial representation of the essential procedures involved in cancer image detection and classification. In the middle of the operation between image acquisition and result production, those operations above must be effectively processed with several calculations.

An automated and efficient model is required for handling the complexities and time consumption in tumor image diagnosis from MRI scans [4]. It is observed from several types of research that soft computing techniques are effectively incorporated for processing. Here, the classification of images is performed with an efficient, gentle computing technique called artificial neural networks. According to the report generated after processing the input MRI, related treatments or therapies are provided by the doctors to the concerned patients. The technique of detection is primarily being developed for the purpose of detecting brain cancers at an earlier stage. The patient's recuperation process may be made more accessible as a result of this. Many different types of researches are being conducted in this area, particularly in the detection and classification of brain tumours, as a result of the rising need for medical or clinical support systems for tumour diagnosis. As a result of this, the primary goal of this study is to build a soft computing technique-based brain tumour diagnostic model, known as APSO (accelerated particle swarm optimization) based artificial neural network model (ANNM), in which preprocessing of MRI images is accomplished by the use of a median filter. Following that, the segmentation process is carried out with the help of FCM, and the feature extraction process is carried out with the help of GLCM. Furthermore, the categorization of MRI is performed using ANN. The stated findings are taken into consideration in a significant way for providing patients with suitable and efficient treatment processes in real-time medical services. The primary goal of the proposed study is to develop an accurate segmentation of brain tumour MRI images using machine learning techniques.

It is necessary to change the brain tumour feature extraction for easier classification. It is also necessary to categorise the tumour pictures using neural network algorithms and neuro-fuzzy algorithms. It is also necessary to segment and identify the brain tumour by combining CT and MRI images. The remaining part of the paper is organized as follows: Section 2 describes the existing models for brain tumor detection and other parts of the body.  Section 3 narrates the working procedure of the proposed soft computing based brain tumor detection and classification (APSO (accelerated particle swarm optimization) based artificial neural network model (ANNM).  Section 4 contains the results and comparative evaluations of the proposed model. Finally, Section 5 presents the conclusion of the work with some enhancement way of the present work.

## 2. Related Works

In [5], segmentation-based brain tumor detection technique has been presented, and the accuracy of the model was determined by comparing with other existing models. In the model, the internal structure has been analyzed by considering the significant factors of tumor detection. An improved tumor approximation of brain cells was presented based on the segmentation process and two-dimensional and three-dimensional visualization for treatment planning and tumor evaluation [6]. The shape approximation of a tumor cell has been effectively designed for treatment patterns.

The work provided by the authors of [7] used the FCM technique to separate the tumor region of interest from the complete brain image. Moreover, the model avoided estimating the members of the FCM group by proper data selection and pixel setting, which are also involved in performing appropriate segmentation of cancer mass. The performance evaluations were carried out based on the significant parameters such as accuracy, precision, sensitivity, and specificity. Further, in work [8], anisotropic filtering has been used for preprocessing the input image, and SVM-based classification technique was used for producing different classification results. With the use of anisotropic filtering, the noise has been effectively removed from the MRI input. After performing morphological operations, the affected part of the brain with the appropriate location has been identified correctly. Moreover, the classifications have been made with the pixel intensities obtained from the filtered MRI inputs for accurate tumor detection.

In [9], a hybrid model has been constructed in which segmentation was done with the OTSU threshold-based technique, and feature extraction was accomplished with morphological operations. The segmented result and the original MRI were compared and assessed to measure the proper detection of the tumor location. *K*-nearest neighbor-based brain tumor detection has been described in [10]. The classifier distance has been assessed using the Manhattan factor. Local binary pattern (LBP) based feature extraction has been employed in [11] for successfully obtaining edges and spots. Moreover, in that work, Gabor features and spectral features were retrieved utilizing two layers of fusion approaches. The collected numerous characteristics were concatenated to achieve appropriate classification results. In [12], the authors have studied two separate frameworks, such as Cascade NN architecture (CASNN) and feed forward NN (FFNN) (FFNN).

Further, feature extraction has been performed using principal component analysis (PCA) to minimize computational complexities. The work used the Olivetti Research Lab (ORL) database data set for evaluations. The training and testing have been carried out using neural network techniques.

In work [13], a hybrid classification technique has been used to classify tumor images that include support vector machine (SVM) and fuzzy logic techniques. The work also incorporated image enhancement methodologies such as stretching the middle range of pictures and contrast improvement. Skull modeling was performed with morphological functions. An ensemble-based classification model has been developed in [14]. The comparisons have been established with 11 individual classifiers, and 36 data sets have been used for analysis. Pruned associative model for cancer detection from obtained clinical images was obtained in [15]. The authors have used CT brain images for testing. And, for earlier identification of brain tumors perceptron-based neural network model (PNN) has been described in [16]. The abnormality of input images has been effectively detected using the region severance technique.

Statistical Association Rule Mining technology has been applied in [17] for effective tumor picture identification. Moreover, coefficient-based weight computations were used for tumor detection. Effective comparison assessments were done in [18] by generating the findings of Close+, Association Rule Mining, and Apriori algorithm-based classifications in medical picture identification. Association rule mining was utilised in [19] for analyzing kidney images for finding the disorders in that. Further, the discretization-based feature extraction technique has been applied in that diagnosis model for reducing the complications in mining the evaluated images.

Further, in the works of [20, 21], association techniques and classification models used for disease diagnosis from medical images have been effectively described. In [22], backpropagation neural networks were used for kidney disease diagnosis. The processing time is not effectively determined and considered by analyzing the existing models in the medical image processed in tumor diagnosis. This paper focuses on developing a model with minima classification errors and processing time for enhancing the precision results on time for assisting the medical practitioners in disease diagnosis [23].

## 3. Proposed Model

For reducing the death rate of cancer patients, the proposed model utilised soft computing techniques for detecting the brain tumor in earlier stages. Moreover, brain tumor detection is carried out using ANN classification from the segmentation of MRI scan images. As in the general tumor detection process, the proposed soft computing-based brain tumor detection and classification (APSO (accelerated particle swarm optimization) based artificial neural network model (ANNM) contains four phases, namely, MRI image preprocessing, segmentation, feature extraction, and classification [24].

The initial preprocessing phase is carried out using a median filter and edge detection to reduce the noise in from the obtained image and clearly define the vision for further process. Following, the images used for segmentation, which is done with fuzzy *C*-means clustering, and the feature extraction process [25] are performed to select appropriate features through which the brain tumor is detected precisely, which is done with GLCM incorporation. After completing all, the filtered images are given to artificial neural networks for classification that performs training and testing effectively. The work process of the proposed model is presented in Figure 2.

### 3.1. Preprocessing

The human brain images are complex and composite in structure, which make the processing complicated. It is required to remove the unwanted noises from the obtained MRI image [26]. Here, the preprocessing phase is carried out using the median filter and edge detection.

#### 3.1.1. Median Filter

Noise elimination from the input MRI images performed with the median filter that uses a non-linear filtering process. This kind of filter is used to remove salt and pepper noise, specifically based on the average pixel rates [27].  Figure 3 presents an MRI brain image results after applying a median filter into that.

#### 3.1.2. Using Edge Detection

Edge detection is utilised here to detect and identify the sharp discontinuities in the MRI image. Here, the Canny edge detection approach is applied for suitable localization of edge points [28]. And, the discovered edge sites utilizing the edge detection model are displayed in Figure 4.

### 3.2. Accelerated Particle Swarm Optimization

Segmentation is a significant process in the tumor detection process that segregates the input image into several regions overlapping each other [29]. It is used to define the object boundaries effectively and the segmented parts are combined to get the full image. The segmentation process is processed based on image intensities that mainly concentrate on the similarity and discontinuity factors of images. There are several available techniques for image segmentation, amongst which fuzzy *c*-means clustering model is used. Here, the FCM method is used for enhancing the precision in image segmentation with an appropriate definition of the object function [30]. Further, the local and nonlocal-based object segmentation is processed by the effective definition of the objective function.

The image of the MRI scan is divided into several pixels [31], which are given as *P*={*p*_1_,  *p*_2_,   … *p*_*n*_}. And, based on the member rate of each pixel, it as belonging to one or more clusters. Several iterations are carried out for reducing the objective function with the member set “*F*” called fuzzy membership, and “*U*” is considered to be the cluster center.

(1) $$\begin{array}{c} Objective\;Function\;\left(A\right)=\overset{n}{\underset{i=1}{\sum }}\overset{U}{\underset{j=i}{\sum }}F_{ij}^{m}{\left(p_{i}-U_{j}\right)}^{2} \end{array}$$

where “*F*_*ij*_^*m*^” denotes the pixel member table, “*m*” is the fuzzy parameter of the cluster, and (*p*_*i*_ − *U*_*j*_) is the Euclidean distance between the pixel member and the cluster center. It is evaluated that point closer to “*U*” has the highest rate of membership than the other points towards the boundaries. In FCM, the cluster centers are initially assigned and rate for each cluster. Then, the center points are shifted to the exact place by increasing the number of iterations based on the data set [27].The data presented in the image and the fuzzy parameter are defined by the pixel member. Further, the pixel member *F*_*ij*_ and cluster center “*U*” are updated based on the defined objective function, which is given as follows:

(2) $$\begin{array}{c} F_{ij}=\frac{1}{\sum_{k-1}^{U}{\left(p_{i}-U_{j}/p_{i}-U_{k}\right)}^{2/m-1}} \end{array}$$

The derivation process will end, when the value reaches *maxi*_*ij*_{|*F*_*ij*_^(*k*+1)^ − *F*_*ij*_^*k*^|} < *α*, where ‘*α*' is the ending factor that lies between 0 and 1. Moreover, the cluster center vector is calculated as

(3) $$\begin{array}{c} U_{j}=\frac{\sum_{i-1}^{n}U_{ij}^{m}p_{i}}{\sum_{i-1}^{n}U_{ij}^{m}} \end{array}$$

The steps in FCM-based segmentation are described below

1. Initialization with cluster center *U* = [*u*_*ij*_] matrix, *U* (0).
2. At *k*^th^ step, the cluster center is calculated as given in (3).
3. The iterations can be terminated at the point it reaches, *maxi*_*ij*_{|*F*_*ij*_^(*k*+1)^ − *F*_*ij*_^*k*^|} < *α*, else, go to step 2.

### 3.3. Gray-Level Co-Occurrence Matrix-Based Feature Extraction

Extracting proper features from the images is a significant process for defining effective classification patterns for précised result categorizations. In this work, the feature extraction process is computed with GLCM, which is an effective arithmetic process that uses the spatial pixel similarities for computations [32]. Based on the pixel intensities of the input images, the spatial similarities between two pixels can be defined as the relationship between the pixel of interest and the adjacent pixel in horizontal positions. For each pixel element (*a*, *b*) in defining GLCM is considered by the number of occurrences of the pixel with “*a*” presented in the described spatial similarity to another pixel with the value “*b*” in the obtained MRI. Moreover, the process is very much helpful in pointing the exact tumor location [33] and its present stage to providing proper treatment assistance.

In this model, the main features considered for evaluation are shape, color, image intensity, texture, contrast, homogeneity, correlation, and energy.

(i) Shape:
As a general definition, shape denotes the geometrical features of an object or its clear edges concerning their composition, color, and image texture.
(ii) Color and Image Intensity:
Here, color is also considered as an important feature, which can be noted by the image coordinates, and the strength of color is denoted as intensity.
(iii) Texture:
The visual quality of the image is noted as texture, which is also derived here.
(iv) Contrast:
Contrast is evaluated by analyzing the separation of lighter and the darker areas in the image as
  (4) $$\begin{array}{c} contrast=\overset{n-1}{\underset{ab=0}{\sum }}p_{ab}{\left(a-b\right)}^{2} \end{array}$$
(v) Homogeneity:
It denotes the closeness of element or object distribution on to the matrix diagonals, which points to the homogeneous quality.
  (5) $$\begin{array}{c} Homogeneity=\overset{n-1}{\underset{ab=0}{\sum }}\frac{p_{ab}}{1+{\left(a-b\right)}^{2}} \end{array}$$
(vi) Correlation:
The correlation coefficients are generally ranged between -1 and +1 and computed as
  (6) $$\begin{array}{c} Corr=\overset{n-1}{\underset{ab=0}{\sum }}p_{ab}\frac{\left(a-\mu \right)\left(b-\mu \right)}{\sigma^{2}} \end{array}$$
(vii) Energy:
Here, energy is defined as the sum of squared pixels rates of the defined gray-level co-occurrence matrix, which is computed as
  (7) $$\begin{array}{c} Energy=\overset{n-1}{\underset{ab=0}{\sum }}{\left(p_{ab}\right)}^{2} \end{array}$$

### 3.4. Artificial Neural Network Model (ANNM) Based Classification

In the proposed work, artificial neural network (ANN) is used for performing the classification operation. This classification technique is incorporated here for its adaptive learning abilities, self- organization pattern, and well suitable nature of real-time implementations. The network pattern contains three layers, input layer, hidden layer, and output layer, which are given in Figure 5.

There are two kinds of operations are performed in ANN, namely, training and testing. In training operation, the neural network is trained with the obtained features that are extracted from the previous section, and testing is performed effectively for validation of results. The parameters that are used for ANN designing are presented in Table 1.

The activation function used here is “purelin” and “tansig” that represent the hyperbolic tangent sigmoid function and linear transfer function. And the learning model used here is Levenberg–Marquardt backpropagation, which is the speed training method. The mean square rate is the computation of the number of errors that occurred in the classification process. Here, the artificial neural network is trained with input MRI images that contain 5 nodes in hidden layer nodes and 1 node at the output layer. The activation functions are applied at the hidden and output layer. After recovering features from the feature extraction procedure, training samples and testing samples are segregated and supplied for testing in ANN and backpropagation technique, respectively. The obtained results are evaluated using the evaluation parameters such as sensitivity, specificity, precision, and accuracy.

## 4. Results and Comparisons

The proposed model is analyzed using the MATLAB tool for implementation with the benchmark data set known as DICOM databases containing MRI brain images [22]. Clinical practitioners develop brain images in the database with different brain modalities. For evaluating the present model, 750 brain samples are considered for training and testing with the artificial neural networks. The results are compared with the existing models to justify the proposed model's accuracy and efficiency [34] in producing outcomes.

For providing evidence for the proposed model, the obtained results are compared with the existing models such as PNN and FCM-based cancer detection. Support vector machine (SVM) and perceptron found neural network model (PNN). Each training and testing phase is processed with 18 brain samples divided into 9 each for training and testing, respectively. The trained representatives are provided as input to the ANN for training, and the validation is carried out with the testing samples. After performing simulations, the value computed for models without tumor is almost similar to 0, and cancer presented images to obtain about 1 and classified based on that. The sample brain images obtained from the Dicom library are shown in Figure 6. The brain images that are diagnosed with tumors after performing 500 iterations are given in Figure 7.

### 4.1. Performance Measures

The performance of the proposed model is measured using metrics such as specificity, sensitivity, and accuracy rates using true-positive, true-negative, false-positive, and false-negative rates. Moreover,

(i) True-positive rate is to evaluate brain images with tumor that are correctly detected as abnormal.
(ii) True negative is defined as the normal samples are mentioned as normal.
(iii) A false positive is the tumorless sample that is falsely identified as containing a tumor.
(iv) False negative in the abnormal samples is incorrectly defined as normal.
(v) Here, sensitivity, specificity, and accuracy rates are computed as
  (8) $$\begin{array}{c} \text{sensitivity}=\frac{\text{true positive}}{\text{true positive}+\text{false negative}}\times 100\\ \text{specificity}=\frac{\text{true negative}}{\text{true negative}+\text{false positive}}\times 100\\ \text{accuracy}=\frac{\text{true positive}+\text{true negative}}{\text{true positive}+\text{true negative}+\text{false positive}+\text{false negative}}\times 100 \end{array}$$

Based on the above factors and computations, the performances of the proposed work in classifying brain tumor images are evaluated.

### 4.2. Comparative Evaluations

When applying the ANN computing for tumor image classifications, the performance is evaluated with the training, testing, and validation results. The performance graph is given in Figure 8 with the assumption of 50 iterations and the minimum mean square error is considered as 10^−5^. At the 19^th^ iteration, the best value is achieved with a minimal error rate of 0.0000041.

The results obtained on accurate classification results are evaluated and portrayed in Figure 9. It is observed from the figure that the proposed APSO (accelerated particle swarm optimization) based artificial neural network model (ANNM) received a better accuracy rate than other classification techniques. The proposed soft computing-based cancer detection model produces a 42% or higher accuracy rate than other classification models. The optimal solution is ensured by the effective integration of segmentation, feature extraction, and classification based on soft computing.

As mentioned in Section 4.1, the performance measures to the derived model are computed and the obtained results are.

They are presented in Figure 10. The obtained results are compared for the existing models, such as PNN and SVM. It can be noted from the figure that the soft computing-based classification model acquired better results than the compared models. The model produces 96% of accuracy in brain tumor detection and classifications. Moreover, the model uses minimal processing time than other models, which is considered a significant factor in evaluating a classification model. In the proposed model, the median filter and edge detection methods are used for preprocessing, making the detection process faster than other methods. It is given in Figure 11. Here, the processing time is estimated against the number of brain images processed over seconds. The comparative evaluations results show the efficiency of the proposed model in producing accurate and précised results with minimal processing time.

Figure 12 represents the training images.  Figure 13 represents the testing images.

The graph on the right illustrates the results of a performance study of brain scans. Listed in Table 2 is a list of the network parameters that were utilised to train the artificial neural network. Comparing the results of the current algorithm with the suggested outcome is shown in the second table.

Table 3 represents the performance metrics. A false-negative diagnosis based on an MRI scan might send the neurologist and patient down the wrong road, causing them to miss an appropriate diagnosis or perhaps postpone it altogether. While MRI is not the sole piece of the jigsaw in the diagnosis of brain tumours, it is an important element of the equation.

Generalizations aside, it is possible to classify data sets into two categories: training data sets and testing data sets. The correctness of the categorization is essentially determined by the two basic procedures, namely the training and testing processes, which are carried out. It is necessary to evaluate a brain tumour classification system when it has been appropriately trained on the largest available database of tumours. Testing the classification system's accuracy in categorising various forms of brain tumours during this phase provides for the verification of the system's correctness. The technique that has been described may be used to more than 70 distinct photographs at the same time. The various MRI brain scans are collected from a local medical facility. In the proposed technique, there has been a significant improvement in the efficacy of its classification.

## 5. Conclusions and Future Enhancement

In the present scenario of medical image processing, an efficient methodology is required for accurate tumor diagnosis. This paper presents a new model using a soft computing technique based on brain tumor detection and classification for assisting the radiologists in providing efficient treatments to the affected persons. Moreover, the median filter is used here for noise removal, and edge detection is used to accurately define the MRI brain image. For segmenting the tumor image effectively, Fuzzy c-means clustering is incorporated. Further, the feature extraction for performing efficient classification is performed with GLCM. The derived features of obtained brain images are given for ANN-based sort, which results in an appropriate type with an accuracy rate of 96.6%. The simulation results show that the proposed work produces better classification results compared to the existing models in terms of metrics such as classification accuracy, error, model efficiency, and processing time.

In the future, the work can be enhanced in such a manner to categorise the stages of the tumor for improving the decision pattern to provide treatments.

## Figures and Tables

**Figure 1:** General functions involved in tumor diagnosis process.

**Figure 2:** Work process of (APSO (accelerated particle swarm optimization) based artificial neural network model (ANNM).

**Figure 3:** Process of applying median filter in MRI brain image: (a) image with noise and (b) image after noise removal.

**Figure 4:** (a) Input image and (b) after edge detection.

**Figure 5:** ANN structure.

**Figure 6:** Sample brain images from DICOM data set.

**Figure 7:** Brian images diagnosed with tumor.

**Figure 8:** Performance analysis graph.

**Figure 9:** Accuracy rate comparisons.

**Figure 10:** Evaluation of methods with performance measures.

**Figure 11:** Processing time comparisons.

**Figure 12:** Training images.

**Figure 13:** Testing images.

**Table 1:** Parameters definition for ANN.

Parameters	Initial values
Activation functions	“Purelin” and “tansig”
Nodes in hidden layer	16
Learning model	Levenberg–Marquadrt backpropagation
Learning rate	0.005
Number of epochs	500
Mean square error	10^–5^
Minimum error	0.002
Momentum rate	0.6
Training time	50 seconds

**Table 2:** Input feature parameters using feature extraction.

Images/features	Mean	Standard deviation	Entropy (bits/pixel)	Contrast	Correlation	Energy
1	1.9280	16.4988	0.0567	0.0689	0.6971	0.3648
2	0.5689	17.3836	0.0697	0.6791	0.8799	0.5678
3	0.3598	16.9167	0.0689	0.0359	0.6946	0.7861
4	0.8857	13.8738	0.0689	0.0264	0.9647	0.6871
5	0.2678	12.4463	0.0698	0.0698	0.9764	0.8674

**Table 3:** Performance metrics comparison

Performance metrics	SVM [23]	Fuzzy logic [18]	Proposed
Accuracy	95.5.	97.68	99.875
Sensitivity	0.97	0.99	0.99
Specificity	0.85	0.90	1.0

## Data Availability

The data that support the findings of this study are available on request from the corresponding author.
